# Augmentation in Healthcare: Augmented Biosignal Using Deep Learning and Tensor Representation

**DOI:** 10.1155/2021/6624764

**Published:** 2021-01-27

**Authors:** Marwa Ibrahim, Mohammad Wedyan, Ryan Alturki, Muazzam A. Khan, Adel Al-Jumaily

**Affiliations:** ^1^Faculty of Engineering and Information Technology, University of Technology Sydney, NSW 2000, Sydney, Australia; ^2^Faculty of Artificial Intelligence, Al-Balqa Applied University, Al-Salt 19117, Jordan; ^3^Department of Information Sciences, College of Computer and Information Systems, Umm Al-Qura University, P.O. Box 715, Makkah, Saudi Arabia; ^4^Department of Computer Science, Quaid-i-Azam University, Islamabad 44000, Pakistan; ^5^School of Computing and Mathematics, Charles Sturt University, Wagga Wagga, Australia; ^6^College of Computing, Fahad Bin Sultan University, Tabuk, Saudi Arabia

## Abstract

In healthcare applications, deep learning is a highly valuable tool. It extracts features from raw data to save time and effort for health practitioners. A deep learning model is capable of learning and extracting the features from raw data by itself without any external intervention. On the other hand, shallow learning feature extraction techniques depend on user experience in selecting a powerful feature extraction algorithm. In this article, we proposed a multistage model that is based on the spectrogram of biosignal. The proposed model provides an appropriate representation of the input raw biosignal that boosts the accuracy of training and testing dataset. In the next stage, smaller datasets are augmented as larger data sets to enhance the accuracy of the classification for biosignal datasets. After that, the augmented dataset is represented in the TensorFlow that provides more services and functionalities, which give more flexibility. The proposed model was compared with different approaches. The results show that the proposed approach is better in terms of testing and training accuracy.

## 1. Introduction

In healthcare systems, data are not publicly available, and these data are limited in nature too. For example, in the current pandemic, the COVID-19, no data are publicly available and some institutes have very limited data [1, 2]. As a result, machine learning and big data analytics cannot be performed on such limited data. One possible solution is to augment limited data and increase the data for testing and training of various machine learning algorithms. The main purpose of Data Augmentation (DA) is to increase the data size [2]. Also, DA is a technique that strongly invades the field of data mining and processing for regression and classification purposes, particularly in healthcare applications. The expression DA denotes the techniques used to generate virtual samples. The created latent samples are introduced to the original data to produce a high-dimensional one. The newly generated augmented data are used in training the suggested model. DA algorithms become numerous. The manipulation between DA algorithms is to achieve high accuracy results and at the same time, implementing modest and rapid algorithm is a typical matter of talent [2]. The appropriately selected DA technique drives the accuracy values to a dramatic level. Researchers developed an approach to combine, search, and select the best augmentation scheme between deterministic, marginal, and conditional different augmentations methodologies. This developed approach was applied to three different classes of systems and achieved good results among these systems [1–3].

Augmentation may be applied in two domains; the first domain is the data domain, while the second one is the feature domain [4]. Many studies demonstrated the art of DA by generating numerous training samples [5]. Other studies focused on the advantage of DA and how it might act as an organizer to prevent associated overfitting during training of neural networks [6] and develop the execution to avoid problems that may be correlated with the classes that are not represented equally [7]. Many researchers prospected in the field of DA to achieve high accuracy values and enhance the classifier performance. A punch of distorted and warped samples of characters are generated by the DA technique [8]. This was not the only example of creating deformed samples of characters as it was reported in [9], where the malformed samples are generated in a random manner. The latter mentioned methodology was extended to be applied on backpropagation neural networks and reduced the error rate to 0.4% on the MNIST database [10]. After that, in [4], the researchers followed two augmentations techniques. The first applied augmentation technique was data wrapping or DA on the input of MNIST dataset before being introduced to neural networks, then the output features from the neural networks were augmented in the feature domain. They used SVM, ELM, and backpropagation neural networks as classifiers, where the accuracy percentage ranged between 97.75% and 100% for training samples.

In the same context, DA was hired by generating virtual samples [11]. Generally speaking, the virtual samples can be generated by following two techniques. The first methodology depends on generating virtual samples from important information. For example, in the field of image processing and recognition, we can generate virtual samples from the same image by producing a 3D view, which in turn helps in creating virtual samples for the same image from a different angle [12].

Consequently, the proposed model has the ability to enhance learning performance, especially when dealing with a few samples. A lot of these mentioned sample generation techniques have shown considerable potential to improve classification and prediction performance. In spite of that, none of the previous studies are built on the overlapping found in the features step. Accordingly, this article presents a new model based on generating a virtual sample that also considers solving overlaps between each of the features in the corresponding classes. Moreover, this model is distinct by its ability to create and treat with a massive amount of new virtual samples that are hundreds of thousands of samples rather than tens or hundreds of virtual samples.

In this article, previous works are presented in Section 2. In Section 3, we illustrated the proposed model that consists of data acquisition, random virtual generation equations, and experiment. Then, in Section 4, we presented and explained the results. Finally, in Section 5, the conclusion and future work are discussed.

## 2. Previous Work

DA was recalled and implemented in many studies. For example, in [13], the researchers established a relation between the iterative computational time for the expectation-maximization procedure and extension of the space parameter with augmenting the data. The recognized relation was an expansion to the applied space parameter applied along with DA, where the iterative computation time was expected to be shorter. Earlier, scientists calculated the posterior probability for the augmented data when the normal likelihood could not be reached [14]. The DA was used in different fields as, for example, in [15] the concept of replicating the data in the field of chemistry. Image recognition was one of the fields where DA took innovative steps, as in [16]. The scholars applied manual augmentation techniques in conjunction with deep neural network that led to an enhanced achievement. Moreover, the experimenters implemented DA algorithm for hand-drawn dataset and a fine-tuned deep neural network to extract useful features from the introduced dataset [17]. Recently, the authors of [18] applied the DA Markov chain Monte Carlo (MCMC). Furthermore, the scholars in [19] applied augmentation in both data domain and feature domain along with using the neural network for an acoustic signal, while in [20], the authors applied augmentation to the speech signal to prove that the gap between real room impulse response and simulated one was reduced to its minimum value. In addition, the authors of [21] combined the deep belief networks and DA algorithm, adding gamma variables to the original signal. In the field of image processing, the scholars augmented the input image by generating a 3D copy to be processed in the neural network [22]. Finally, researchers in [23] applied the augmentation and balancing to the electroencephalography (EEG) signal.

On the other hand, the tensor representation was used in different research fields to allow for a better representation of the dataset. In 20th century, scientists paid attention to the value of tensors and their applications [24]. In the field of continuum mechanics, tensor fundamentals and enforcement were discussed [25]. A study addressed the tensor decomposition technique [26] and treated it as a generalization for matrix decay. In [27], the concept of deep tensor neural network (DTNN) was initially introduced where one of the layers was substituted by a double projection layer. Those two inserted are totally nonlinear. Therefore, any input vocabulary speech was mapped to the newly introduced in conjunction with a tensor layer. The model was capable of anticipating the next layer in the deep neural network design. The proposed model resulted in reducing error by 3% relatively. The researchers in [26] and in [28] developed a model that was able to estimate an approximation for tensor rank 1 by disintegrating tensor and estimating Canonical Polyadic Decomposition (CPD) by using a sparse matrix of the banded type. In 2014, the inequality of the M tensors was discussed in [29], where the upper and lower values for the eigenvalues were obtained. In [30], the authors demonstrated the modeling of earthquake waveform to estimate the moment tensor solution. The estimation of tensor parameters was deeply analyzed in [31]. Furthermore, tensor decomposition techniques were presented in [32] to give the opportunity for a more latent dataset than that based on the matrix domain. Recently, in [33], the authors applied the tensor decomposition on the genetic expression to a group of latent components used to find a relation between any biological development and genetic variation.

In [34] to increase the accuracy of the soft sensor under the small sample issue, they proposed a new locally linear embedding based virtual sample generation approach. In the proposed approach, the first step is producing features from the original data space by using locally linear embedding. The next step is generating effective virtual samples in the sparse region of the original data by using a method of random interpolation and a backpropagation neural network. To test the performance of the proposed approach, a couple of studies were conducted: the first study is a process of high-density polyethylene and the second study is developing soft sensors for a production system of purified terephthalic acid. The outcomes showed that the precision with virtual samples improved for the soft sensor. Moreover, the proposed method achieved more accuracy than other approaches in virtual sample generation.

Finally, in [35], the study simulated the process of fishermen rectifying nets; this method was named Kriging-VSG and it was put forward to produce feasible virtual samples in data-sparse zones. This method was based on a distance-based criterion by imposing each dimension to recognize important samples with huge data gaps. Similar to the procedure of fishermen rectifying nets, a specific dimension was fixed at various quantiles. The numerical simulations and a real-world application from a cascade reaction process for high-density polyethylene were achieved to check the performance of the proposed method. The performance was superior to other methods.

## 3. The Proposed Model

This section shows detailed steps to explain the model we developed in this work, from data acquisition to the generation of the virtual samples required and from constructing the model to the classification tool.

### 3.1. Data Acquisition

Our proposed model was examined on different datasets. The two datasets are classified into finger movements and the UCI machine learning respiratory. The first dataset was recorded by implementing two surface channels by using FlexComp device. The sensors were of type T9503M and were positioned on the patient forearm, as shown in Figure 1.

Nine participants were asked to perform ten finger movements. Each finger movement consumed five seconds, then there was a rest for another five seconds, and then the participant was requested to execute the next finger movement and so on till finishing the ten finger movement classes, which are shown in Figure 2. The mentioned data collection process were repeated for six times.

The second dataset was for amputee patients. The nine participants missed their left hand. The goal of collecting these data was to classify between six different gestures to understand and analyze the controlled upper limbs prostheses. The six gestures were flexion, index flexion, fine pinch, tripod grip, hook grip, and spherical grip. It was a very challenging task to record the surface signal from amputee participants with three different force levels. The skin was cleaned with alcohol and prepared using the abrasive method. The allocated electrodes were Ag/AgCl electrodes.

The surface signal was recorded from 8 channels at three levels of forces for nine amputee participants. The first dataset was amplified by 1000; the first and second datasets were sampled at 2000 Hz.  Figure 3 shows the allocation of the electrodes and the collection of the surface signal from amputee participants.

For the above-mentioned datasets, threefold cross-validation was applied, where 2/3 of dataset was assigned to the training set, whereas 1/3 was allocated to the testing set. The data were filtered to secure the precision and removal of noise. The training and testing accuracies were estimated on average basis where the accuracy was calculated per subject and the overall accuracy was the summation of each accuracy per subject divided by the number of subjects.

Other datasets were imported from UCI machine learning respiratory, which was considered as a strong archive that was cited more than 1000 times by machine learning community researchers. The performance of the proposed model was observed on additional five datasets that were archived at the UCI website. Those multiclass datasets were Iris, Breast Cancer, Seeds, Sonar, Mines vs. Rocks, and Indian Liver Patient. The Iris dataset is one of the most popular datasets that has been implemented in the pattern recognition field. The Iris dataset had three classes: one class was linearly independent of the other two classes and could be easily separated, whereas the other two classes were not separable. The three targeted classes for Iris dataset were Iris setosa, Iris virginica, and Iris versicolor. The Breast Cancer dataset was collected from the doctor clinic and classified into six classes, of which two were benign and the other four classes were dedicated for malignant type. The dataset was collected for three different sorts of wheat. The three different classes for the seeds dataset were Kama, Rosa, and Canadian, which were recorded via X-ray plates. The Sonar, Mines vs. Rocks dataset was to discriminate between metal and rock. The last recalled dataset was Indian Liver Patient. The dataset was collected from 441 male Indian participants and 142 female participants to discriminate if this participant could be classified as a liver patient or not.

### 3.2. Random Virtual Generation Equations

Let us assume that we have dataset *e*=(*x*, *f*(*x*)), where *e* represents the original training samples, *x*  ∈  *R*_*n*_, and *f*(*x*)={−1,  1}. Assume that we have previous information *k*, and we need to map our training set to the new domain. Therefore, if we have a convert that equals *T*= *y*_*T*_, the dataset *e* will be transformed via this conversion equation to generate virtual samples (*Tx*,  *y*_*T*_(*f*(*x*)). The generation of mathematical transformation *T* and *y*_*T*_ depends primarily on the previous information, which may result in either simple or complex transformation formula.

However, the second algorithm depends on adding noise to the original signal [36]. Most of the techniques that were used to create virtual samples suffer from the lack of combining reasonableness and adaptability simultaneously. Accordingly, we followed an algorithm to generate virtual Gaussian samples [2]. This method started to calculate the mean and standard deviation for Gaussian distribution, as shown in Figure 4. Then, the virtual samples could be generated following this technique, and finally, the virtual generated samples were added to the original ones [37]. So, { *x*_1_,…*x*_*n*_, *x*_*n*+1_,…*x*_*k*_} represents the original dataset, which belongs to *R*. The first *n* samples of the dataset are continuous, whereas the *k* − *n* samples are discrete. The *m* random variables are generated by Gaussian algorithm *N*=(*μ*,  *η*^2^) for the first *n* continuous samples knowing that *μ* represents the mean and *η* represents the standard error. However, for the samples *k* − *n* that are assigned to be discrete ones, the values will not be transformed and in order to keep the consistency between the discrete and continuous part, we may generate random variables for the discrete part by using *N*=(*μ*,  *η*^2^) with *η*^2^ equalling zero. Figure 1 shows the normal distribution for augmented data for one feature only. This technique was utilized in our proposed model, where the main motivation was to secure a normal distribution for the stochastic electromyography signal.

The tensor can be defined as a multidimensional array with respect to a basis; however, for a vector, it can be represented as a single-dimensional array with respect to the same basis. In brief, tensors can be evaluated as a multidimensional vector. Tensors can be deemed as a mathematical method to represent values in a multidimension matrix. Tensors are considered the comprehensive version of matrix, vector, and scalar. Therefore, matrix, vector, and scalar can be measured as subcomponents of tensor. The generation of tensor can be done by following transformation laws. Tensors are characterized as having various coordinate systems. Therefore, the coordinate systems with their transformation laws will be analyzed in the next section.

Assume that we have *x*^*i*^, where *i*=1,2,…, *N*. So, by substituting the different values of *i*, we can get *N*  values of *x* in a *N*-dimensional space *x*^1^, *x*^2^,…, *x*^*N*^. Moreover, the set of ${\bar{x}}^{i}$ can be expressed as ${\bar{x}}^{1},\;{\bar{x}}^{2},\ldots ,{\bar{x}}^{N}$ for *N*-dimensional coordinates. In the same context, keeping the same transformation laws for *x*′ to ${\bar{x}}^{\prime }$ leads to the following transformation equation:

(1) $$\begin{array}{c} x^{i}=\;x^{i}\;\left({\bar{x}}^{1},\;{\bar{x}}^{2},\ldots {\bar{x}}^{N}\right),\;i=1,2,\ldots ,N. \end{array}$$

The above equation creates an independent relation between the two different coordinates *x*^*i*^ and ${\bar{x}}^{i}$ for *i*=1,2,…, *N*. As long as the relation is kept independent, it can be recalled for transformation.

The Jacobian first-order partial transformation will be estimated as follows:

(2) $$\begin{array}{c} J\left(\frac{x}{\bar{x}}\right)=J\left(\frac{x^{1},x^{2},\ldots ,x^{N}}{{\bar{x}}^{1},\;{\bar{x}}^{2},\ldots ,{\bar{x}}^{N}}\right)=\;\left|\begin{array}{cccc} \frac{\partial x^{1}}{\partial {\bar{x}}^{1}} & \frac{\partial x^{1}}{\partial {\bar{x}}^{2}} & \ldots & \frac{\partial x^{1}}{\partial {\bar{x}}^{N}}\\ \vdots & \vdots & \cdots & \vdots \\ \frac{\partial x^{N}}{\partial {\bar{x}}^{1}} & \frac{\partial x^{N}}{\partial {\bar{x}}^{2}} & \cdots & \frac{\partial x^{N}}{\partial {\bar{x}}^{N}} \end{array}\right|. \end{array}$$

With an inverse transformation,

(3) $$\begin{array}{c} {\bar{x}}^{i}={\bar{x}}^{i}\left(\;x^{1},x^{2},\ldots ..,x^{N}\right),\;i=1,2,\ldots ,N. \end{array}$$

In brief, both equations (1) and (2) can be expressed in the notation formula as follows:

(4) $$\begin{array}{c} x^{i}=\;x^{i}\;\left(\bar{x}\right),\;i=1,2,\ldots ,N, \end{array}$$

(5) $$\begin{array}{c} {\bar{x}}^{i}={\bar{x}}^{i}\left(x\right),\;i=1,2,\ldots ,N. \end{array}$$

$\bar{x}$ can be concluded from *x* and $\bar{\bar{x}}$ can be deduced from $\bar{x}$ by recalling transformation. Assume that $\bar{x}=y$ and $\bar{\bar{x}}=z$ . The transformations are represented by *T*_1_, *T*_2_, and *T*_3_, where

(6) $$\begin{array}{c} T_{1}:y^{i}=\;y^{i}\left(x^{1},\;x^{2},\ldots ,x^{N}\right),\;i=1,2,\ldots ,N\text{ or }T_{1}x=y,\\ T_{2}:z^{i}=\;z^{i}\left(y^{1},\;y^{2},\ldots ,y^{N}\right),\;i=1,2,\ldots ,N\text{ or }T_{2}y=z. \end{array}$$

*T*_3_ can be deduced by the product of both *T*_1_ and *T*_2_:

(7) $$\begin{array}{c} T_{3}:z^{i}=\;z^{i}\left(y^{1}\left(x^{1},\;x^{2},\ldots ,x^{N}\right),\ldots ,y^{N}\left(x^{1},\;x^{2},\ldots ,x^{N}\right)\right),\;i=1,2,\ldots ,N\\ \text{or }T_{3}x=T_{2}T_{1}x=z\text{ by considering }T_{3}=T_{2}T_{1}, \end{array}$$

where *T*_1_, *T*_2_, and *T*_3_ represent the first, second, and third coordinates transformations, respectively.

## 4. Experiment

The study implemented two layers of autoencoder: the first layer was 1200 nodes, whereas the second was 900 nodes. The encoder transfer function was purely linear. The suggested model is shown in Figure 5.

We claimed that the suggested paradigm was able to achieve high accuracy values for both the training and the testing sets with a powerful signal representation. In a preparatory step of the model, the input raw biosignal was performed by algorithm. The implemented window size was 200 milliseconds, while window increment was 50 milliseconds. The recommended number of sampling points to calculate the discrete Fourier transform was 1024. The advantage of proceeding lies in providing an appreciated representation for the input raw biosignal, which, in turn, boosted the accuracy values for both training and testing set. The output of representation was fed to the DA stage, where the above-mentioned Gaussian augmentation was used with reiterating represented data 1000 times. Reiterating data 1000 times was followed based on different trials, where 1000 showed the most compromise between simulation time and performance. The DA enriched the data and granted affluence to the data that improved training and testing accuracies in return. As a final stage in representing data, the tensor representation was hired to give us the opportunity to demonstrate the data into a developed perspective. Then, the data was presented to two layers of autoencoder to learn features from high-quality represented data. The first layer of autoencoder was 1200 nodes, whereas the second one was 900 nodes.

The weight regularization coefficient was set to 0.001, as its default value, for both layers of autoencoder. The coefficient that controlled the weights of the sparsity regularization was set to 4 for both layers. The sparsity proportion factor determined the activation response rate of the autoencoder neuron. The value of sparsity proportion varied from 0 to 1. A lower value promoted and inspired for a higher sparsity. The sparsity proportion was set to 0.05. Eventually, the encoder transfer function was set to purely linear. We executed different transfer functions like logistic and positive saturating linear transfer functions aside from the pure linear one, which led to promoted results. The output features were employed to proceed with the classifier phase. The paper used three different main classifiers, namely, ELM, SVM, and SL. In terms of ELM, five activation functions were used and picked out the activation function that generated the most precise results. The five executed activation functions, namely, Sine, Triangular basis, and Radial basis functions. As for the SVM classifier, the study proceeded with six different functions for SVM. The executed SVM functions were linear, quadratic, cubic, fine Gaussian, medium Gaussian, and coarse Gaussian SVM, and the function that performed the best outcome was selected. The accuracies of the three classifiers were presented to the classifier fusion layer to select the best local classifier per class.

## 5. Results

The implementation of the classifier layer endorsed the accuracies for both training and testing set as the training set. The classification accuracy of ten finger movements dataset accounted for 100% for the training pack and 90.25% for testing one. As for the high-force six finger movements dataset, the training collection accuracy amounted to 99.74%, whereas accuracy for the testing group achieved 91.85%. Then, the executed data representation techniques mentioned above and the deep neural network were replaced by a typical pattern recognition model where the features were extracted and reduced to a lower number of features by using linear discriminant analysis and that used both the ELM and the SVM as classifiers. However, the performance of the ELM as a classifier was much better than that achieved by the SVM in terms of both the simulation time and accuracy. Based on the used pattern recognition model, the training accuracy for ten finger movements was 95.76%, whereas testing accuracy was 87.11%, as illustrated in Figure 6. In terms of the six finger movements, both the training and the testing accuracies were lower than those values achieved by our proposed model. The training accuracy was 98.57%, whereas the testing one was 89.64%, as illustrated in Figure 7.

This study concluded that our proposed model was explicitly better than the typical pattern recognition model. Furthermore, the suggested system did not require any feature as it was trained to learn features by itself and independent of the input data. Accordingly, we examined the planned scheme on popular datasets to provide the model with reliability and trustworthiness. The implementation of Iris data resulted in a training accuracy of 100 % and testing accuracy of 98.5%. For Breast Cancer tissue dataset, the training accuracy was 98.58% and testing accuracy was 91.7%. However, using Sonar dataset, the accuracy for training was 85.69% and that for testing was 74.4%. Moreover, executing liver dataset led to 96.47% as training accuracy and 85.1% for testing one. With regard to the data, the training accuracy accounted for 94.57%, whereas for testing one, it amounted to 83.6%. The UCI machine learning respiratory datasets were executed without recalling any classifier fusion layer and were classified by using classifier only. The training simulation time was more than 600 seconds. However, the time consumed for examining the testing set on the trained network was not more than 1.5 seconds.  Table 1 shows both training and testing accuracies for all of the above-mentioned datasets. Figure 6 shows a comparison between the testing and the training accuracies for the suggested model and those resulted from implementing a typical pattern recognition technique for classifying the ten finger movements. However, Figure 7 shows the same comparison for the six finger movements. The recommended model did not only show better performance on the level of training and testing accuracies but also saved the effort and time that might be wasted in selecting the best features that match the application.

## 6. Conclusion and Future Work

We suggested a deep learning model where the data were represented, augmented, and then transferred into the tensor domain. Two layers of autoencoder were implemented by adjusting its parameters to have the best results. The SVM, ELM, and SL were applied as classifiers. Also, the best local classifier was applied to select the highest accuracy per class. The proposed model was applied to different datasets to provide it with fidelity and reliability. Ten and six finger movements were used for the advised system and for traditional pattern recognition. The planned diaphragm resulted in higher accuracies than the traditional pattern recognition system with the advantage of the classifier fusion technique. Moreover, the pattern recognition consumed effort and time to extract the best features set that led to better accuracies, whereas the suggested model did not require any features or human interventions as it was capable of learning features by itself regardless of the introduced dataset. The recommended model consumed about 600 seconds to train the network with no more than 1.5 seconds to test the trained network. The planned model was applied to other popular datasets and brought about accepted accuracy values. The main advantage behind examining data by the model was that we voided the feature extraction engineering handcrafted techniques and fed the model by the data that were capable of learning features by itself and independently of the data type that was introduced, which saved time and effort. Eventually, as a future enhancement, the simulation time may be reduced by implementing different neural networks that may be able to learn features in a superior manner without consuming a long simulation time.

## Figures and Tables

**Figure 1:** Posture of the electrodes.

**Figure 2:** Ten different finger gestures (classes).

**Figure 3:** Electrodes allocation for amputee participants.

**Figure 4:** The normal distribution for one feature after DA [1, 2].

**Figure 5:** Proposed model diagram.

**Figure 6:** Comparison between suggested deep learning model in ten finger movements.

**Figure 7:** Comparison between suggested deep learning model in six finger movements.

**Table 1:** Training and testing accuracies for all implemented datasets.

Dataset	Training accuracy (%)	Testing accuracy (%)
Ten finger movements (suggested deep learning model)	100	90.25
Six finger movements (suggested deep learning model)	99.74	91.85.
Ten finger movements (typical pattern recognition)	95.76	87.11
Six finger movements (typical pattern recognition)	98.57	89.64
Iris (suggested deep learning model)	100	98.5
Breast tissue (suggested deep learning model)	98.58	91.7
Sonar (suggested deep learning model)	85.69	74.4
Seeds (suggested deep learning model)	94.57	83.6
Liver (suggested deep learning model)	96.47	85.1

## Data Availability

The data used to support the findings of this study are available from the corresponding author upon request.
